# Fusion of Hsp70 to Mage-a1 enhances the potency of vaccine-specific immune responses

**DOI:** 10.1186/1479-5876-11-300

**Published:** 2013-12-05

**Authors:** Juhong Jiang, Dan Xie, Wenmin Zhang, Gang Xiao, Jianming Wen

**Affiliations:** 1 Department of Pathology, The First Affiliated Hospital, Guangzhou Medical University, 151, Yanjiang Road, Guangzhou 510120, China; 2 State Key Laboratory of Oncology in South China, Cancer Center, Sun Yat-Sen University, 651# Dongfeng Road East, Guangzhou 510060, China; 3 Department of Pathology, Fujian Medical University, 88, Jiao Tong Road, Fuzhou, Fujian 350004, China; 4 Department of Pathology, Kiang Wu Hospital, Macau, China; 5 Department of Pathology, The First Affiliated Hospital, Sun Yat-sen University, 58, Zhongshan Road II, Guangzhou 510080, China

**Keywords:** Mage-a1, Heat-shock protein 70, Protein vaccine, Humoral immunity, Cytotoxic T lymphocyte

## Abstract

**Background:**

Heat shock proteins (HSPs) are capable of promoting antigen presentation of chaperoned peptides through interactions with receptors on antigen presenting cells. This property of HSPs suggests a potential function as an adjuvant-free carrier to stimulate immune responses against a covalently linked fusion partner. MAGE-A1 is a likely candidate for tumor immunotherapy due to its abundant immunogenic epitopes and strict tumor specificity. To analyze the influence of HSP70 conjugation to MAGE-A1, towards developing a novel effective vaccine against MAGE-expressing tumors, we cloned the murine counterpart of the human HSP70 and MAGE-A1 genes.

**Methods:**

Recombinant proteins expressing Mage-a1 (aa 118–219), Hsp70, and Mage-a1-Hsp70 fusion were purified and used to immunize C57BL/6 mice. The humoral and cellular responses elicited against Mage-a1 were measured by ELISA, IFN-γ ELISPOT assay, and cytotoxicity assay.

**Results:**

Immunization of mice with Mage-a1-Hsp70 fusion protein elicited significantly higher Mage-a1-specific antibody titers than immunization with either Mage-a1 alone or a combination of Mage-a1 + Hsp70. The frequency of IFN-γ-producing cells and the cytotoxic T lymphocyte (CTL) activity was also elevated. Consistent with the elevated immune response, immunization with fusion protein induced potent *in vivo* antitumor immunity against MAGE-a1-expressing tumors.

**Conclusions:**

These results indicate that the fusion of Hsp70 to Mage-a1 can enhance immune responses and anti-tumor effects against Mage-a1-expressing tumors. Fusion of HSP70 to a tumor antigen may greatly enhance the potency of protein vaccines and can potentially be applied to other cancer systems with known tumor-specific antigens. These findings provide a scientific basis for the development of a novel HSP70 and MAGE fusion protein vaccine against MAGE-expressing tumors.

## Background

The molecular cloning of MAGE-1 by van der Bruggen et al. in 1991 provided a major breakthrough in identifying tumor antigens recognized by host cytotoxic T-lymphocytes (CTL). Using the melanoma cell line MZ2-MEL and autologous CTL clones cytolytic to this line, MAGE-1 (subsequently re-named MAGE-A1/melanoma antigen A1) was identified as the target antigen for one of the CTL clones, representing the first immunogenic tumor antigen shown to elicit autologous CTL responses in a cancer patient [1]. Subsequent studies showed that MAGE-A1 is a member of a family (the MAGE gene family) encoding proteins that are classified as tumor antigens, also referred to as cancer testis (CT) antigens. These antigens are expressed by tumors of different histological types, but are silenced in normal cells (with the exception of the male germ-line cells of the testis, which do not express MHC class I molecules and are therefore incapable of presenting antigens to CTLs). More than 100 CT antigen family proteins have now been identified, and some of these have been shown to be capable of eliciting immune responses [2]. Because CT antigens are immunogenic and their expression is highly restricted to tumors, they represent an ideal target for tumor immunotherapy.

Tumor vaccines derived from MAGE-A1 have been used in several small–scale phase I/II therapeutic vaccination trials. Patients with advanced malignancies of cutaneous melanoma, non–small-cell lung cancer (NSCLC) or head and neck, esophageal, or bladder cancer were enrolled in these trials. These trials consisted of antigenic peptides, protein, recombinant poxvirus-encoding mini-genes, or dendritic cells (DCs) pulsed with antigenic peptide. No significant toxicity was reported; however, only a small proportion of the patients (10 to 20%) showed evidence of tumor regression [3-7]. Therefore, it is important to develop a more potent MAGE-A1-based vaccine.

The combined use of heat shock proteins (HSPs) has been explored as a strategy for enhancing vaccine potency [8-15]. HSPs are a large family that includes inducible and also ubiquitously and constitutively expressed protein chaperones [10]. The effect of HSPs on immunotherapy was first indicated by the demonstration that HSPs purified from tumor cells, but not normal tissues, can immunize animals to generate tumor-specific immunity. The immunogenicity of the tumor-derived HSPs was shown to be dependent on the peptides associated with HSP molecules rather than the HSPs *per se*[11].

HSP-based cancer vaccines, including tumor-derived HSP-peptide complex, artificially reconstituted HSP-peptide complex, HSP-based DNA cancer vaccines, and HSP fusion protein, have been widely explored in tumor models [12]. Among these HSP preparations in different formulations, the fusion protein strategy, which allows covalent linkage of multiple antigenic epitopes to a single HSP fusion protein, has been shown to be successful, simple and feasible. The adjuvant property of mycobacterial HSP70 fusion protein has been extensively studied using HIV-1 p24 [13], ovalbumin [14], influenza nucleoprotein [15], MAGE-1 [8] and MAGE-3 [9] as model antigens. In the latter two studies [8,9], a fusion protein linking *Mycobacterium tuberculosis* HSP70 and a human MAGE was used to elicit anti-tumor effects against a mouse melanoma cell line, B16, which was transfected into mice. Although the HSP70-MAGE fusion proteins elicited stronger cellular and humoral immune responses against MAGE-expressing tumors than those elicited by MAGE protein alone, the specificity of the response could be of concern. The use of Mycobacterial HSP70 as an adjuvant in a murine model could elicit cross-reaction with host HSP and thereby induce inappropriate autoimmune responses, including autoimmune-mediated intestinal inflammation [16,17]. Additionally, there are likely to be differences in the processing and presentation of human epitope peptides by the murine MHC system in this model. Thus, the combination of proteins from different species may impart a level of complexity in interpreting the results. To eliminate the risk of inducing autoimmune disorders and to reflect a more authentic murine immune response to tumor antigens, in this study the murine counterpart of the human HSP70 and MAGE-A1 genes (designated Hsp70 and Mage-a1) were cloned. Prokaryotic plasmids were constructed to express a Mage-a1 (aa 118–219) gene segment, Hsp70, and the Mage-a1-Hsp70 fusion protein. The recombinant proteins were expressed and purified for immunization of mice. We demonstrate that linkage of Hsp70 to Mage-a1 enhances the immunogenicity of Mage-a1, which results in increased antitumor humoral and cellular immunity against Mage-a1-expressing murine melanoma cells.

## Materials and methods

### Construction of prokaryotic protein expression vectors

The sequences of the *Mus musculus* Hsp70 and Mage-a1 genes [GenBank: NM_010479 and NM_020015] were used as references for primer design. Forward Primer (5’-*gaattc*gccaagaacacggcgatcggcat-3’ and reverse primer 5’-*gtcgac*aatccacctcctcgatggtgggt-3’) flanked respectively by *Eco*R1 and *Sal*1 restriction sites (italics) were used to amplify the coding sequence for the 2^nd^ to the last amino acid of the Hsp70 gene. Forward Primer (5’- *ggatcc*accaaagcagaaatgttggaaag-3’) and reverse primer (5’- *gaattc*accacacaatcctatgttattca -3’) flanked respectively by *Bam*H1and *Eco*R1 restriction sites (italics) were used to amplify the coding sequence of the Mage-a1gene segment (aa 118–219). DNA extracted from liver tissue of a C57BL/6 mouse was used as template to amplify the Hsp70 and Mage-a1 genes. The PCR products of the two segments were first cloned separately into pGEM-T vector (Promega, USA). After verification by sequencing, recombinant pGEM-T vectors were digested with restriction enzymes, and the isolated segments were separately cloned into pGEX4T-1 to construct pGEX4T-1-Hsp70 and pGEX4T-1-Mage-a1 expression vectors. Then, the Mage-a1 segment was inserted into *Bam*H1- and *Eco*R1-digested pGEX4T-1-Hsp70 vector to obtain the Mage-a1 (aa 118–219)/Hsp70 fusion protein expression vector, pGEX4T-1-Mage-a1-Hsp70. All recombinant expression vectors were verified by sequencing.

### Protein expression and purification

The pGEX4T-1, pGEX4T-1-Mage-a1, pGEX4T-1-Hsp70 and pGEX4T-1-Mage-a1-Hsp70 constructs were transformed into *E. coli* Rosetta 2 (DE3) (Novagen, USA). Bacterial cultures were grown to OD600 ≈ 0.5, and then protein expression was induced by adding 0.1 mM isopropyl β-thiogalactopyranoside (IPTG) to the growth media. Bacteria were cultured at 32°C for 4 hours and then harvested by centrifugation. Cell pellets were resuspended in PBS (4.3 mM Na_2_HPO_4_, 1.47 mM KH_2_PO_4_, 137 mM NaCl, and 2.7 mM KCl, pH 7.3) and stored frozen at −20°C. Upon purification, the suspension was thawed at room temperature. NP-40 was added to the cell suspension at a final concentration of 0.1%, and lysozyme was added at a final concentration of 45 kU/gram of cell paste. Cell pellets were sonicated to suspend thoroughly and shear the DNA. The tubes were centrifuged at high speed to precipitate the cellular debris while leaving the soluble protein in the supernatant. As the target proteins have a glutathione S-transferase (GST) tag, the GST · Band Kit (Novagen, USA), an affinity chromatography column with GST Binding Resin was used to purify the proteins according to the manufacturer's instructions.

### Cell lines

Cells were maintained in RPMI 1640 medium supplemented with 10% fetal bovine serum, 100 mg/ml of streptomycin, and 100 U/ml of penicillin in a humidified atmosphere at 37°C with 5% CO_2_. A murine melanoma cell line B16 was used to generate the B16-Mage-a1 cell line, which stably expresses the *Mus musculus* Mage-a1 gene. To establish the B16-Mage-a1 cell line, the eukaryotic expression vector pcDNA3.1-Mage-a1 was constructed and transfected into B16 cells. Transfected cells were grown in medium containing 600 μg/ml G418 (Sigma, USA) until single colonies appeared. The expression of Mage-a1 in B16-Mage-a1 was determined by RT-PCR (data not shown).

### Mice and vaccination

C57BL/6 mice were obtained from the laboratory animal center of Sun Yat-Sen University (Guangzhou, China). All of the mice were 6 week old females bred and maintained under specific pathogen-free conditions. Purified GST, Hsp70, Mage-a1, Mage-a1-Hsp70 fusion protein, or a combination of Mage-a1 + Hsp70 proteins, were diluted to 200 pmol. Six groups of mice were immunized sub-cutaneously with 0.2 ml of each protein or PBS control, followed by a booster after 1 week. All the procedures are in accordance with the guidelines of the laboratory animal ethics committee of Sun Yat-sen University.

### Anti-Mage-a1 ELISA

Anti-Mage-a1 antibody in the sera of vaccinated mice was determined by ELISA. Briefly, a 96-well flat-bottom ELISA plate was coated with 50 μl of 2.5 μg/ml Mage-a1 protein (aa 118–219) overnight at room temperature. The plate was rinsed with PBS, incubated with blocking buffer (5% nonfat dry milk powder and 0.2% Tween 20 in PBS) for 2 h at 37°C. Mouse serum was diluted 1:50 in blocking buffer, added to the plate, and incubated for 2 h at 37°C. After rinsing with PBS, the plate was incubated with horseradish peroxidase-conjugated anti-mouse IgG (Santa Cruz Biotech Inc., USA) for 1 h at 37°C. After extensive washing, Tetramethyl-benzidine substrate was added, and plates were incubated for 20 min at room temperature. The reactions were stopped with 2 M H_2_SO_4_, and the ELISA plates were read at 450 nm.

### IFN-γ ELISPOT

Mice were sacrificed two weeks after the immunization booster was injected. Splenocytes were isolated using EZ-Sep Mouse 1X Lymphocyte Separation Medium (Dakewe, China) according to the manufacturer's instructions. IFN-γ production of T cell precursors was determined by using the Quick Spot Mouse IFN-γ Pre-coated ELISPOT kit (Dakewe, China) according to the manufacturer's instructions. PVDF-bottomed 96-well plates were pre-coated with anti-IFN-γ antibody. A total of 200 μl of RPMI 1640 was added to each well, plates were incubated for 10 min, and then medium was removed. 5 × 10^5^ splenocytes/well and 3 × 10^4^ B16-Mage-a1 cells/well were added. As a positive control, 5 × 10^4^ splenocytes/well and 4 μg/ml phytohemagglutinin (PHA) were added. As a negative control, only serum-free culture medium was added. Plates were incubated without agitation for 24 h at 37°C. Cells were then removed and biotinylated IFN-γ detection antibody was added and plates were incubated for 1 h at 37°C. Free antibody was washed out, and plates were incubated with streptavidinalkaline phosphatase for 1 h at 37°C, followed by 10 washes with PBST and visualization with alkaline phosphatase substrate AEC. The number of dots in each well was counted using Biosys Bioreader 4000 PRO (Bio-sys, German). The experiment was repeated three times.

### Cytotoxicity assays

The Cytotoxic 96 nonradioactive cytotoxicity assay (Promega, USA) was used to detect the cytotoxic activity of splenocytes from mice immunized with the protein vaccines. This assay quantitatively measures lactate dehydrogenase (LDH), a stable cytosolic enzyme that is released upon cell lysis. To develop the effector cells, splenocytes isolated as in the ELISPOT assay were co-cultured with lethally irradiated (10000 rad of ^60^Co) B16-Mage-a1 cells in the presence of 40 U/ml rhIL-2 (Cytolab Ltd./Peprotech Asia, USA) for 3 days at 37°C. According the manufacturer's instructions, we first optimized the number of B16-Mage-a1 target cells at 1 × 10^4^ and then set up the 96 well assay plate. In the experimental wells, effector cells at a ratio of 1:2.5, 1:5, and 1:10 were added to 1 × 10^4^ target cells to a final volume of 200 μl. The plate was incubated for 45 min at 37°C and centrifuged at 500 g for 5 min. Subsequently, 50 μl supernatant from each well was transferred to a new plate, and 50 μl substrate mix was added to each well. The plate was incubated for 30 min at room temperature in darkness. A total of 50 μl stop solution was added to each well, and the absorbance values were measured at 490 nm. The cytotoxicity for each effector: target cell ratio was calculated as [A(experimental)-A(effector spontaneous)-A(target spontaneous)] × 100%/[A(target maximum)-A(target spontaneous)].

### In vivo mouse tumor challenge

For inoculation of tumor cells, cultured cells were collected and washed twice in serum-free RPMI 1640. Viable cells were counted using trypan blue and a cell meter. Cell suspensions were adjusted to a concentration of 1 × 10^6^ cells/ml, and 0.1 ml cell suspension was inoculated sub-cutaneously in the upper flank of mice. For tumor protection experiments, 6 groups of mice were immunized with GST, Hsp70, Mage-a1, Mage-a1 + Hsp70, Mage-a1-Hsp70 or the PBS control, followed by a booster after one week. One week after the booster, mice were challenged with 1 × 10^5^ B16-Mage-a1 cells/mouse. For *in vivo* tumor treatment experiments, another 6 groups of mice were first challenged with 1 × 10^5^ B16-Mage-a1 cells/mouse. At 3 days and 10 days post-tumor cell inoculation, mice were immunized. Tumor growth was observed every day. Tumor length and width were measured at fixed time intervals. The tumor volume was defined as V (V = length × width^2^ × 0.5), where V represents the mean value of tumors in each group. Mice were sacrificed when the tumor length reached 15 mm.

### Statistical analysis

All statistical analyses were carried out using Graphpad Prism 5 software for Windows. Results are presented as mean ± standard error (SE). Data were analyzed by one-way analysis of variance (ANOVA) and two-way ANOVA. P values < 0.05 were considered statistically significant.

## Results

### Expression and purification of recombinant proteins

To determine whether fusion of Mage-a1 to Hsp70 can increase the potency of vaccination against Mage-expressing tumors, we expressed *Mus musculus* Mage-a1, Hsp70, and Mage-a1-Hsp70 fusion proteins using the prokaryotic expression vector pGEX4T1, which produces GST-tagged recombinant proteins (Figure 1A). Only part of the Mage-a1 coding sequence (aa 118–219) was cloned because full length Mage-a1 failed to produce detectable protein after IPTG induction. High level protein expression was induced by IPTG for the control pGEX4T1 vector and the three GST tagged vectors in *E. coli* Rosetta 2 (DE3) cells, and the proteins were purified by GST affinity chromatography (Figure 1B-D). A single predominate band of expected size of the purified protein was isolated for each of these proteins, though additional faint bands could be observed in each purification, indicating that some level of degradation or contamination may have occurred. In an attempt to remove the GST tag of the recombinant protein before use in the vaccine experiment, we digested the proteins with thrombin; however, recombinant Hsp70 protein was cut to several bands after thrombin digestion, potentially due to nonspecific thrombin cleavage recognition sites in the Hsp70 sequence (data not shown). Therefore, the GST tags in the recombinant proteins were not removed, and instead, a GST control group was added to our experiments to exclude the effects of the GST tag or common contaminants.

**Figure 1:** **Construction of vectors and recombinant protein expression and purification. A**. Schematic representation of recombinant pGEX4T1 vectors. Mage-a1 (aa118-219) gene segment, Hsp70 and Mage-a1-Hsp70 fusion gene were cloned into pGEX4T1 vector downstream of the GST sequence. **B**. GST protein was expressed by the vector pGEX4T-1 in *E. coli* Rosetta 2. M, protein molecular weight markers. Lanes 1–2, whole cell lysate without and with IPTG induction. Lane 3, purified GST protein. **C**. Mage-a1 protein expressed by recombinant vector pGEX4T-1-Mage-a1. M, protein molecular weight markers. Lanes 1–2, whole cell lysate without and with IPTG induction. Lanes 3–4, purified Mage-a1 protein at 2× or 1× loading concentration. **D**. Hsp70 and Mage-a1-Hsp70 protein expressed by recombinant vector pGEX4T-1-Hsp70 and pGEX4T-1-Mage-a1-Hsp70. M, protein molecular weight markers. Lanes 1–2, whole cell lysate of *E. coli* Rosetta 2 transformed with pGEX4T-1-Hsp70 without and with IPTG induction. Lanes 3–4, purified Hsp70 protein at 1× or 2× loading concentration. Lanes 5–6, whole cell lysate of *E. coli* Rosetta 2 transformed with pGEX4T-1-Mage-a1-Hsp70 without and with IPTG induction. Lanes 7–8, purified Mage-a1-Hsp70 protein at 1× or 2× loading concentration.

### Enhanced induction of Mage-a1-specific humoral immune responses by fusion of Mage-a1 with Hsp70

To examine the immune response elicited by the purified proteins, six groups of mice were injected sub-cutaneously with GST, Hsp70, Mage-a1, Mage-a1-Hsp70 or Mage-a1 + Hsp70 (1:1 mixture). Mice were also injected with 0.2 ml PBS as an additional control. One week later, a booster vaccine was administered, and two weeks after the booster, the quantity of anti-Mage-a1 antibody in the sera of the vaccinated mice was determined by ELISA. Mice vaccinated with PBS control, GST and Hsp70 proteins showed low or undetectable levels of anti Mage-a1 antibody. In contrast, mice vaccinated with Mage-a1, Mage-a1 + Hsp70, and Mage-a1-Hsp70 had elevated levels of anti-Mage-a1 antibody. Of these three, the mice vaccinated with Mage-a1-Hsp70 fusion protein produced the highest levels of anti-Mage-a1 antibody (Figure 2). These results verify that Mage-a1 fusion to Hsp70 leads to an elevated humoral immune response against Mage-a1.

**Figure 2:** **Humoral immune response after vaccination with Hsp70-Mage-a1 fusion protein.** Purified GST, Hsp70, Mage-a1, Mage-a1-Hsp70 fusion protein or a combination of Mage-a1 + Hsp70, were diluted to a concentration of 200 pmol. Mice were immunized sub-cutaneously with a PBS control or 0.2 ml of each protein, followed by a booster injection after one week. Serum samples were obtained two weeks after the booster. The levels of anti-Mage-a1 antibody were examined by ELISA. The means ± SE of the absorbance (A540 nm) of three separate experiments are presented at 1:50 dilution. Statistical analysis by one-way ANOVA showed that mice vaccinated with Mage-a1-Hsp70 had significantly higher titers of anti Mage-a1 antibody than Mage-a1 or Mage-a1 + Hsp70 (* p < 0.001).

### Enhanced induction of T-cell-mediated Mage-a1-specific immune responses by fusion of Mage-a1 with Hsp70

To determine whether mice can induce T-cell-mediated Mage-a1-specific immune responses after vaccination with Mage-a1-Hsp70, mice were immunized and the splenocytes were harvested and pooled two weeks after administration of the booster. B16-Mage-a1-specific IFN-γ production of T cell precursors was determined by ELISPOT assay, which is a sensitive functional assay used for the identification and enumeration of cytokine-producing cells at the single cell level. As shown in Figure 3A, very few spot-forming T cell precursors were observed in the splenocytes from mice injected with PBS, GST or Hsp70 control proteins. However, there were many more spot-forming T cell precursors in the splenocytes from mice injected with Mage-a1, Mage-a1 + Hsp70, and Mage-a1-Hsp70 fusion protein. Moreover, the number of spot-forming cells in the Mage-a1-Hsp70 group was higher than the Mage-a1 and Mage-a1 + Hsp70 groups. This result suggests that Mage-a1 can elicit B16-Mage-a1-specific IFN-γ production by splenic T cell precursors, but that the Mage-a1-Hsp70 fusion protein has a stronger effect than Mage-a1 alone or Mage-a1 separately combined with Hsp70.

**Figure 3:** **T-cell-mediated immune response after vaccination with Hsp70-Mage-a1 fusion protein.** C57BL/6 mice were immunized with purified GST, Hsp70, Mage-a1, Mage-a1-Hsp70 fusion protein or Mage-a1 + Hsp70 and then administered a booster immunization after one week. Two weeks after the booster, pooled splenocyte cultures were prepared and re-stimulated. **A**. IFN-γ-producing T cells in splenocytes of immunized mice were quantified by using ELISPOT. Data are presented as mean ± SE of three separate experiments. Statistical analysis by one-way ANOVA revealed that mice vaccinated with Mage-a1-Hsp70 generated more IFN-γ spots than Mage-a1 or Mage-a1 + Hsp70 (* p < 0.001). **B**. The CTL response induced in splenocytes of immunized mice was determined by using CytoTox 96 nonradioactive cytotoxicity assay. Data are presented as mean ± SE of three separate experiments. Statistical analysis by two-way ANOVA revealed that Mag-a1-specific lysis of CTLs from mice vaccinated with Mage-a1-Hsp70 was higher than those vaccinated with Mage-a1 or Mage-a1 + Hsp70 at all effector: target cell ratios (* p < 0.001).

To assess whether B16-Mage-a1-specific CTLs are induced in immunized mice, splenocytes were also assesses by cytotoxicity assay. Effector cells were obtained by co-culture of splenocytes with lethally irradiated B16-Mage-a1 cells at increasing ratios. As shown in Figure 3B. The percentage of CTLs undergoing B16-Mage-a1-specific lysis was less than 10% in splenocytes from mice injected with PBS control, GST and Hsp70 proteins. However, splenocytes from mice injected with Mage-a1, Mage-a1 + Hsp70 and Mage-a1-Hsp70 showed higher levels of lysis than the controls. Furthermore, the Mage-a1-Hsp70 group promoted more CTL lysis than the Mage-a1 and Mage-a1 + Hsp70 groups. Together, these results suggest that Mage-a1 vaccine can induce Mage-a1-specific T-cell-mediated immune responses and that the fusion of Mage-a1 with Hsp70 protein can enhance this effect.

### Prophylactic immunization with the Mage-a1-Hsp70 fusion protein confers protection against Mage-a1-expressing tumors

To further verify the immune response induced by Mage-a1-Hsp70 fusion protein, *in vivo* tumor protection was investigated in C57BL/6 mice. One week after the booster, mice were challenged with B16-Mage-a1 cells. The PBS control mice and mice vaccinated with GST and Hsp70 proteins developed measureable tumors starting at 13 days after the tumor cell challenge (Figure 4A). However, 100% of mice vaccinated with the Mage-a1-Hsp70 fusion protein remained tumor-free until 19 days after challenge, whereas mice vaccinated with Mage-a1 and Mage-a1 + Hsp70 remained tumor-free until 16 days after challenge. Mage-a1 containing vaccines also induced a significant growth repression for tumors that developed subsequently, with Mage-a1-Hsp70 fusion protein showing a stronger effect than Mage-a1 and Mage-a1 + Hsp70 (Figure 4B). Therefore, Mage-a1-Hsp70 fusion protein both delays the development of tumors and represses the growth of Mage-a1-expressing tumors in vaccinated mice.

**Figure 4:** **Prophylactic immunization with Mage-a1-Hsp70 fusion protein protects mice against B16-Mage-a1 tumor cell challenge.** C57BL/6 mice were immunized with purified GST, Hsp70, Mage-a1, Mage-a1-Hsp70 fusion protein or Mage-a1 + Hsp70 and then administered a booster immunization after one week. A week after the booster, the mice were challenged with 1 × 10^5^ B16-Mage-a1 melanoma cells. **A**. The tumor free status of mice was recorded as the percentage of mice remaining tumor-free every three days after tumor challenge. **B**. Tumor growth was recorded as the mean tumor volume (in mm^3^). Error bars depict the SE, n = 8 mice/group. Statistical analysis by two-way ANOVA revealed that from days 31 to 37 vaccination with Mage-a1-Hsp70 significantly delayed tumor growth in the B16-Mage-a1 tumor model compared to vaccination with Mage-a1 or Mage-a1 + Hsp70 (* p < 0.01).

### Therapeutic immunization with the Mage-a1-Hsp70 fusion protein confers protection against the progression of established tumors

Given that immunization of mice with the Mage-a1-Hsp70 fusion protein conferred protection against challenge with B16-Mage-a1 cells, we further investigated whether immunization with Mage-a1-Hsp70 fusion protein could block the progression of pre-established tumors. C57BL/6 mice were injected with 1 × 10^5^ B16-Mage-a1 cells. At 3 and 10 days post-tumor cell inoculation, mice were immunized, and tumor development was assessed every 3 days thereafter. The mice vaccinated with PBS, GST or Hsp70 control proteins developed tumors starting at 13 days after the tumor cell challenge (Figure 5A). However, 100% of mice receiving Mage-a1-Hsp70 fusion protein vaccination remained tumor-free 16 days after the tumor cell challenge, whereas only 62.5% and 75% mice receiving Mage-a1 and Mage-a1 + Hsp70 vaccination remained tumor-free. The tumor growth also was repressed in mice vaccinated with Mage-a1, Mage-a1-Hsp70 and Mage-a1 + Hsp70 compared to vaccination with PBS and the other control proteins (Figure 5B), though the effect was not as dramatic as for the prophylactic immunization (Figure 4B). Nevertheless, these results suggest that the Mage-a1-Hsp70 fusion protein has protective effects both for prophylactic and therapeutic immunization against Mage-a1-expressing tumors in mice.

**Figure 5:** **Therapeutic immunization with the Mage-a1-Hsp70 fusion protein confers protection against the progression of established tumors.** Mice were challenged with 1 × 10^5^ B16-Mage-a1 cells. At 3 and 10 days post-tumor cell inoculation, mice were immunized with purified GST, Hsp70, Mage-a1, Mage-a1-Hsp70 fusion protein or a combination of Mage-a1 + Hsp70. **A**. The tumor free status of mice was recorded as the percentage of mice remaining tumor free after tumor challenge. **B**. Tumor growth was recorded as the mean tumor volume (in mm^3^). Error bars depict the SE, n = 8 mice/group. Statistical analysis by two-way ANOVA revealed that vaccination with Mage-a1-Hsp70 significantly delayed tumor growth in the B16-Mage-a1 tumor model compared to vaccination with Mage-a1 or Mage-a1 + Hsp70 from days 31 to 37 (* p < 0.05).

## Discussion

Because the MAGE-A1 antigens are shared by many tumors and because of their strict tumor specificity, they are of particular interest for cancer immunotherapy. The MAGE-A1 gene encodes several antigenic peptides that bind to HLA class I or class II molecules and are recognized by T lymphocytes on tumor cells [18-20]. These antigens have been used for small-scale therapeutic vaccination trials of cancer patients [3-7]. However, generally, the induced immune response is weak, necessitating the development of other immunization approaches to increase the efficacy of the vaccines.

Heat shock proteins have demonstrated increasingly more effective use as adjuvants in the immunotherapy of malignant tumors and infectious diseases. Antigen fusion with hsp70 has proven powerful as a strategy to increase the immunogenicity of a conjugated protein [9,13-15]. To study the adjuvant property of HSP70 fusion in enhancing a MAGE-A1-based vaccine in a preclinical mouse model, we constructed prokaryotic plasmids and expressed and purified recombinant Mage-a1, Hsp70, and Mage-a1-Hsp70 fusion proteins. The choice of using Mage-a1-Hsp70 recombinant fusion protein for immunization was based on several theoretical advantages over vaccines consisting of commonly used “short” peptides. First, after being taken up, processed, and presented by professional APCs, Mage-a1 long proteins are much more likely to elicit an integrated immune response consisting of a variety of CD4+, CD8+, and B cell responses [21,22]. Second, it is likely that protein vaccination leads to the presentation of epitopes that can be presented by a variety of HLA alleles, and therefore this type of vaccine should be applicable to any patient regardless of HLA restriction. In addition, the fused Hsp70 protein can activate professional antigen-presenting cells (APCs) and cross-present chaperoned antigenic peptides to MHC class I molecules to generate specific cytotoxic T-lymphocytes [23].

The fusion proteins were purified to high homogeneity; however, faint lower molecular weight bands in each purification reaction suggests a possibility that some effects may be due to degraded recombinant proteins, or possibly contaminants. However, the addition of several controls, including PBS alone, vector alone, and each protein either alone or purified separately and then combined, provides verification of our results. Furthermore, our results are consistent with two other studies involving HSP70-MAGE fusions of mixed species origin [8,9]. In the latter studies a fusion protein composed of *Mycobacterium tuberculosis*-derived HSP70 (MtHSP70) and human-derived MAGE was injected into mice; whereas this study tested a fusion protein composed of murine Hsp70 and murine Mage-a1 in mice. The use of a same-species proteins may be advantageous for several reasons: first, the use of murine-derived protein in a mouse model may reduce the risk of inducing autoimmune disease; second, the affinity of murine-derived Hsp70 to Hsp70 receptors on mouse DCs is likely to be higher than the corresponding affinity of MtHSP70; and third, the murine MHC system may more effectively process and present epitope peptides of murine tumor antigens than antigens from human tumors. Therefore, our study both confirms and extends the previous findings by providing a more authentic model.

After the mice were immunized with the protein vaccine, we observed both humoral and cellular immune responses. The humoral response was determined by measuring the quantity of anti-Mage-a1 antibody in the sera of vaccinated mice. The cellular response was determined by measuring B16-Mage-a1-specific IFN-γ production by T cell precursors and B16-Mage-a1-specific CTLs from splenocytes of immunized mice. We demonstrated that mice immunized with GST, Hsp70 protein or PBS control have low or undetectable levels of anti-Mage-a1 antibody in sera, minimal IFN-γ production of T cell precursors from splenocytes, and low-level activation of B16-Mage-a1-specific CTL lysis. Compared with GST, Hsp70 protein or PBS controls, vaccination with Mage-a1, Mage-a1 + Hsp70, and Mage-a1-Hsp70 fusion protein enhanced both the humoral and cellular response, as indicated by elevated serum Mage-a1-specific antibody, increased Mage-a1-specific IFN-γ production and CTL cytotoxicity. Moreover, Mage-a1-Hsp70 fusion protein vaccine induced a more dramatic response than Mage-a1 or Mage-a1 + Hsp70. Though the effect of fusion was more obvious for the cellular response than for the humoral response, it is likely that an interplay between these two immune responses contributes to the vaccine efficacy of Mage-a1-Hsp70. Similar to our findings with Mage-a1, fusion of murine Hsp70 with Hantaan virus nucleocapsid protein (HTNV NP) enhances both the humoral and cellular response to the HTNV NP, but the effects on the cellular response are more obvious [24]. Further study is needed to determine the relative contribution of the humoral response to the efficacy of the Mage-a1-Hsp70 vaccine.

Consistent with the immune responses, *in vivo* tumor protection by vaccination was demonstrated by prophylactic immunization. B16 tumor xenografts in mice immunized with Mage-a1, Mage-a1 + Hsp70, and Mage-a1-Hsp70 fusion protein grew significantly slower than that in mice immunized with GST, Hsp70 protein or PBS control. The tumor size of mice immunized with Mage-a1-Hsp70 fusion protein was also much smaller than that of Mage-a1 and Mage-a1 + Hsp70-immunized mice. In addition, we demonstrated that therapeutic immunization can delay the progression of established tumors, though this effect was decreased compared with the prophylactic immunization. This result suggests that Mage-a1-Hsp70 fusion protein is more proficient at inhibiting tumor development when used earlier in the progression of cancer, suggesting a preferential application for using this vaccine to prevent tumor recurrence in postoperative cancer patients.

The pro-immune effects of HSPs may be related to their molecular properties as intracellular stress proteins. In addition to their involvement in the degradation pathway of cellular proteins during stress condition, HSPs facilitate the correct folding of newly synthesized proteins and are also directly involved in the translocation of proteins across membranes into different cellular compartments [11,25-27]. After exiting the cell and entering the extracellular environment, peptides chaperoned by heat shock proteins can be taken up by antigen-presenting cells (APCs), such as macrophages and DCs. In the cytosol, the associated peptides are cross-presented via endogenous MHC class-I and exogenous MHC class-II pathways [28-30]. Several receptors for HSPs, have been described on APCs, such as CD14 [31], CD40 [32,33], CD91 [34-36], C-type lectin family scavenger receptor A (SR-A) [37], Lox-1 [38] and the Toll-like receptors (TLRs) 2 and 4 [39]. Binding of HSPs to these receptors could promote the maturation and activation of DCs by stimulating DCs to express MHC class II molecules or to secrete cytokines and chemokines [33,40]. As a consequence of the dual function of this chaperone-peptide presentation on MHC class-I and -II molecules, as well as its adjuvant property, efficient peptide-specific T-cell stimulation is achieved. Antigen-HSP70 fusion proteins can generate specific CD8+ T cells responses independent of CD4+ T cell help [41,42]. A possible mechanism for this ability is the activation of DCs to release proinflammatory cytokines, as well as the intrinsic molecular chaperone function of HSP70. Endogenous IL-2 also probably plays an important role in this process. These functions of HSPs may explain the enhanced potency of Mage-a1 when fused to Hsp70.

MAGE-A1 is expressed in diverse histological types of primary and metastatic tumors, such as melanoma, bladder, breast, prostate, and non-small cell lung cancers [43]. The expression on tumors of most histological origins supports the use of the MAGE-A1-HSP70 fusion protein in vaccines for a wide range of cancers expressing MAGE-A1. The strict tumor specificity of this antigen should minimize the damage to normal tissues following immunization. In addition, several MAGE-A1 epitopes recognized by T cells have been identified. Those epitopes can be presented by HLA-A1, A2, A3, A68, B37, B7, B35, B37, B53, and B57, making MAGE-A1-HSP70 fusion protein vaccine available for most (up to 87%) of the HLA types [18-20,44].

The MAGE-A family consists of several subtypes, including MAGE-A1 to MAGE-A12. Although they are expressed by many histologically different neoplasias, individual MAGE-A expression varies among tumor types [45]. However, the theoretical frequency by which cancer cells express at least one of the MAGE-A antigens is reported to be very high [46,47]. Because we have successfully produced a Mage-a1 and Hsp70 fusion protein vaccine and have demonstrated the efficacy of this strategy in increasing the anti tumor immunogenicity against Mage-a1-expressing tumors, we can apply this strategy to other subtypes of MAGE-A to expand the number of patients eligible for MAGE-A and HSP70 fusion protein immunotherapy. To reach an optimal anti-tumor effect for cancer patients, a mixed vaccine with multiple MAGE-A-HSP70 fusion proteins will be desirable.

## Conclusions

In summary, our results indicate that Mage-a1-Hsp70 fusion protein can elicit stronger Mage-a1-specific immune responses and antitumor effects against Mage-a1-expressing tumor than Mage-a1 alone or a combination of Mage-a1 + Hsp70. Thus, HSP70 fusion represents a novel and potentially promising strategy to design MAGE-based vaccines for achieving protective immunity against malignant tumors that express MAGE antigen.

## Abbreviations

HSPs: Heat shock proteins; CT: Cancer testis; CTL: Cytotoxic T lymphocyte; GST: Glutathione S-transferase; DC: Dendritic cells; APC: Antigen-presenting cells; ELISA: Enzyme-linked immunosorbent assay; ELISPOT: Enzyme-linked immunosorbent spot; HLA: Human leukocyte antigen; MHC: Major histocompatibility complex.

## Competing interests

The authors declare that they have no competing interests.

## Authors’ contributions

DX and JW carried out and coordinated the study. JJ, WZ and GX performed the experiments. All authors read and approved the final manuscript.

## References

[B1] Re van der BruggenPTraversariCChomezPLurquinCDe PlaenEVan den EyndeBKnuthABoonTA gene encoding an antigen recognized by cytolytic T lymphocytes on a human melanomaScience19911150381643164710.1126/science.18407031840703

[B2] CTDatabase[(http://www.cta.lncc.br/index.php)]

[B3] van BarenNBonnetMCDrénoBKhammariADorvalTPiperno-NeumannSLiénardDSpeiserDMarchandMBrichardVGEscudierBNégrierSDietrichPYMaraninchiDOsantoSMeyerRGRitterGMoingeonPTartagliaJvan der BruggenPCouliePGBoonTTumoral and immunologic response after vaccination of melanoma patients with an ALVAC virus encoding MAGE antigens recognized by T cellsJ Clin Oncol200511359008902110.1200/JCO.2005.08.37516061912

[B4] SlingluffCLJrPetroniGROlsonWCzarkowskiAGroshWWSmolkinMChianese-BullockKANeesePYDeaconDHNailCMerrillPFinkRPattersonJWRehmPKHelper T-cell responses and clinical activity of a melanoma vaccine with multiple peptides from MAGE and melanocytic differentiation antigensJ Clin Oncol200811304973498010.1200/JCO.2008.17.316118809608PMC2652084

[B5] MackensenAHerbstBChenJLKöhlerGNoppenCHerrWSpagnoliGCCerundoloVLindemannAPhase I study in melanoma patients of a vaccine with peptide-pulsed dendritic cells generated in vitro from CD34 (+) hematopoietic progenitor cellsInt J Cancer200011338539210.1002/(SICI)1097-0215(20000501)86:3<385::AID-IJC13>3.0.CO;2-T10760827

[B6] Chianese-BullockKAPressleyJGarbeeCHibbittsSMurphyCYamshchikovGPetroniGRBissonetteEANeesePYGroshWWMerrillPFinkRWoodsonEMWiernaszCJPattersonJWSlingluffCLJrMAGE-A1-, MAGE-A10-, and gp100-derived peptides are immunogenic when combined with granulocyte-macrophage colony-stimulating factor and montanide ISA-51 adjuvant and administered as part of a multipeptide vaccine for melanomaJ Immunol2005115308030861572852310.4049/jimmunol.174.5.3080

[B7] AkiyamaYTanosakiRInoueNShimadaMHotateYYamamotoAYamazakiNKawashimaINukayaITakesakoKMaruyamaKTakaueYYamaguchiKClinical response in Japanese metastatic melanoma patients treated with peptide cocktail-pulsed dendritic cellsJ Transl Med2005111410.1186/1479-5876-3-415676080PMC549033

[B8] YeJChenGSSongHPLiZSHuangYYQuPSunYJZhangXMSuiYFHeat shock protein 70/MAGE-1 tumor vaccine can enhance the potency of MAGE-1-specific cellular immune responses in vivoCancer Immunol Immunother20041198258341512723710.1007/s00262-004-0536-6PMC11034208

[B9] MaJHSuiYFYeJHuangYYLiZSChenGSQuPSongHPZhangXMHeat shock protein 70/MAGE-3 fusion protein vaccine can enhance cellular and humoral immune responses to MAGE-3 in vivoCancer Immunol Immunother200511990791410.1007/s00262-004-0660-315756604PMC11034288

[B10] FederMEHofmannGEHeat-shock proteins, molecular chaperones, and the stress response: evolutionary and ecological physiologyAnnu Rev Physiol19991124328210.1146/annurev.physiol.61.1.24310099689

[B11] UdonoHSrivastavaPKHeat shock protein 70-associated peptides elicit specific cancer immunityJ Exp Med19931141391139610.1084/jem.178.4.13918376942PMC2191193

[B12] BinderRJHeat shock protein vaccines: from bench to bedsideInt Rev Immunol2006115–63533751716978010.1080/08830180600992480

[B13] SuzueKYoungRAAdjuvant-free hsp70 fusion protein system elicits humoral and cellular immune responses to HIV-1 p24J Immunol19961128738798543845

[B14] MizukamiSKajiwaraCIshikawaHKatayamaIYuiKUdonoHBoth CD4+ and CD8+ T cell epitopes fused to heat shock cognate protein 70 (hsc70) can function to eradicate tumorsCancer Sci20081151008101510.1111/j.1349-7006.2008.00788.x18341654PMC11160078

[B15] AnthonyLSWuHSweetHTurnnirCBouxLJMizzenLAPriming of CD8+ CTL effector cells in mice by immunization with a stress protein-influenza virus nucleoprotein fusion moleculeVaccine199911437338310.1016/S0264-410X(98)00199-69987177

[B16] RaskaMWeiglEHeat shock proteins in autoimmune diseasesBiomed Pap Med Fac Univ Palacky Olomouc Czech Repub20051124324910.5507/bp.2005.03316601763

[B17] SteinhoffUBrinkmannVKlemmUAichelePSeilerPBrandtUBlandPWPrinzIZügelUKaufmannSHAutoimmune intestinal pathology induced by hsp60-specific CD8 T cellsImmunity19991134935810.1016/S1074-7613(00)80110-710514013

[B18] PascoloSSchirleMGückelBDumreseTStummSKayserSMorisAWallwienerDRammenseeHGStevanovicSA MAGE-A1 HLA-A A*0201 epitope identified by mass spectrometryCancer Res200111104072407711358828

[B19] LuitenRvan der BruggenPA MAGE-A1 peptide is recognized on HLA-B7 human tumors by cytolytic T lymphocytesTissue Antigens200011214915210.1034/j.1399-0039.2000.550206.x10746786

[B20] LuitenRMDemotteNTineJvan der BruggenPA MAGE-A1 peptide presented to cytolytic T lymphocytes by both HLA-B35 and HLA-A1 moleculesTissue Antigens2000111778110.1034/j.1399-0039.2000.560110.x10958359

[B21] ZwavelingSFerreira MotaSCNoutaJJohnsonMLipfordGBOffringaRvan der BurgSHMeliefCJEstablished human papillomavirus type 16-expressing tumors are effectively eradicated following vaccination with long peptidesJ Immunol20021113503581207726410.4049/jimmunol.169.1.350

[B22] AtanackovicDAltorkiNKCaoYRitterEFerraraCARitterGHoffmanEWBokemeyerCOldLJGnjaticSBooster vaccination of cancer patients with MAGE-A3 protein reveals long-term immunological memory or tolerance depending on primingProc Natl Acad Sci USA20081151650165510.1073/pnas.070714010418216244PMC2234199

[B23] BendzHRuhlandSCPandyaMJHainzlORiegelsbergerSBraüchleCMayerMPBuchnerJIsselsRDNoessnerEHuman heat shock protein 70 enhances tumor antigen presentation through complex formation and intracellular antigen delivery without innate immune signalingJ Biol Chem20071143316883170210.1074/jbc.M70412920017684010

[B24] LiJLiKNGaoJCuiJHLiuYFYangSJHeat shock protein 70 fused to or complexed with hantavirus nucleocapsid protein significantly enhances specific humoral and cellular immune responses in C57BL/6 miceVaccine200811253175318710.1016/j.vaccine.2008.02.06618479786

[B25] PilonMSchekmanRProtein translocation: how Hsp70 pulls it offCell199911667968210.1016/S0092-8674(00)80780-110380919

[B26] JensenREJohnsonAEProtein translocation: is Hsp70 pulling my chain?Curr Biol19991120R779R78210.1016/S0960-9822(00)80012-310531024

[B27] MorimotoRIKlineMPBimstonDNCottoJJThe heat-shock response: regulation and function of heat-shock proteins and molecular chaperonesEssays Biochem19971117299493008

[B28] BinderRJBlachereNESrivastavaPKHeat shock protein-chaperoned peptides but not free peptides introduced into the cytosol are presented efficiently by major histocompatibility complex I moleculesJ Biol Chem20011120171631717110.1074/jbc.M01154720011278929

[B29] CastellinoFBoucherPEEichelbergKMayhewMRothmanJEHoughtonANGermainRNReceptor-mediated uptake of antigen/heat shock protein complexes results in major histocompatibility complex class I antigen presentation via two distinct processing pathwaysJ Exp Med200011111957196410.1084/jem.191.11.195710839810PMC2213527

[B30] Arnold-SchildDHanauDSpehnerDSchmidCRammenseeHGde la SalleHSchildHCutting edge: receptor-mediated endocytosis of heat shock proteins by professional antigen-presenting cellsJ Immunol19991173757376010201889

[B31] AseaAKraeftSKKurt-JonesEAStevensonMAChenLBFinbergRWKooGCCalderwoodSKHSP70 stimulates cytokine production through a CD14-dependant pathway, demonstrating its dual role as a chaperone and cytokineNat Med200011443544210.1038/7469710742151

[B32] BeckerTHartlFUWielandFCD40, an extracellular receptor for binding and uptake of Hsp70-peptide complexesJ Cell Biol20021171277128510.1083/jcb.20020808312356871PMC2173242

[B33] WangYKellyCGKarttunenJTWhittallTLehnerPJDuncanLMacAryPYounsonJSSinghMOehlmannWChengGBergmeierLLehnerTCD40 is a cellular receptor mediating mycobacterial heat shock protein 70 stimulation of CC-chemokinesImmunity200111697198310.1016/S1074-7613(01)00242-411754818

[B34] BinderRJHanDKSrivastavaPKCD91: a receptor for heat shock protein gp96Nat Immunol200011215115510.1038/7783511248808

[B35] BasuSBinderRJRamalingamTSrivastavaPKCD91 is a common receptor for heat shock proteins gp96, hsp90, hsp70, and calreticulinImmunity200111330331310.1016/S1074-7613(01)00111-X11290339

[B36] FischerNHaugMKwokWWKalbacherHWernetDDanneckerGEHolzerUInvolvement of CD91 and scavenger receptors in Hsp70-facilitated activation of human antigenspecific CD4+ memory T cellsEur J Immunol201011498699710.1002/eji.20093973820101615

[B37] BerwinBHartJPRiceSGassCPizzoSVPostSRNicchittaCVScavenger receptor-A mediates gp96/GRP94 and calreticulin internalization by antigen-presenting cellsEMBO J200311226127613610.1093/emboj/cdg57214609958PMC275431

[B38] MatsutakeTSawamuraTSrivastavaPKHigh efficiency CD91- and LOX-1-mediated re-presentation of gp96-chaperoned peptides by MHC II moleculesCancer Immun201011720672796PMC2964010

[B39] VabulasRMBraedelSHilfNSingh-JasujaHHerterSAhmad-NejadPKirschningCJDa CostaCRammenseeHGWagnerHSchildHThe endoplasmic reticulum-resident heat shock protein Gp96 activates dendritic cells via the Toll-like receptor 2/4 pathwayJ Biol Chem20021123208472085310.1074/jbc.M20042520011912201

[B40] ChenTGuoJHanCYangMCaoXHeat shock protein 70, released from heat-stressed tumor cells, initiates antitumor immunity by inducing tumor cell chemokine production and activating dendritic cells via TLR4 pathwayJ Immunol2009113144914591915549210.4049/jimmunol.182.3.1449

[B41] ZongJPengQWangQZhangTFanDXuXHuman HSP70 and modified HPV16 E7 fusion DNA vaccine induces enhanced specific CD8+ T cell responses and anti-tumor effectsOncol Rep2009119539611972487810.3892/or_00000522

[B42] ChenCHWangTLHungCFYangYYoungRAPardollDMWuTCEnhancement of DNA vaccine potency by linkage of antigen gene to an HSP70 geneCancer Res2000111035104210706121

[B43] CTDatabase[http://www.cta.lncc.br/modelo.php?idgene=11&idmeta=15]

[B44] CTDatabase[http://www.cta.lncc.br/modelo.php?idgene=11&idmeta=6]

[B45] ParkJWKwonTKKimIHSohnSSKimYSKimCIBaeOSLeeKSLeeKDLeeCSChangHKChoeBKAhnSYJeonCHA new strategy for the diagnosis of MAGE-expressing cancersJ Immunol Methods2002111–279861213362410.1016/s0022-1759(02)00105-9

[B46] EuraMOgiKChikamatsuKLeeKDNakanoKMasuyamaKItohKIshikawaTExpression of the MAGE gene family in human head-and-neck squamous-cell carcinomasInt J Cancer199511530430810.1002/ijc.29106405047591301

[B47] OtteMZafrakasMRiethdorfLPichlmeierULöningTJänickeFPantelKMAGE-A gene expression pattern in primary breast cancerCancer Res200111186682668711559535

